# Intelligent Three-Dimensional Reconstruction Algorithm-Based Ultrasound-Guided Nerve Block in Intraoperative Anesthesia and Postoperative Analgesia of Orthopedic Surgery

**DOI:** 10.1155/2022/9447649

**Published:** 2022-07-22

**Authors:** Cuijie Liu, Lin Li, Xuan Zhou, Xiuyan Wang

**Affiliations:** Department of Anesthesiology, Affiliated Hongqi Hospital of Mudanjiang Medical University, Mudanjiang, 157011 Heilongjiang, China

## Abstract

This research was aimed at analyzing the role of ultrasound-guided nerve block based on intelligent three-dimensional (3D) reconstruction algorithm in intraoperative anesthesia and postoperative analgesia of orthopedic surgery. 68 elderly patients were undergoing orthopedic surgery on the lower extremities, and they were randomly rolled into two groups with 34 patients in each group. The patients in control group received sciatic nerve block anesthesia (SNBA), and the patients in the experimental group received ultrasound-guided SNBA (UG-SNBA) under 3D reconstruction algorithm to analyze and compare the anesthesia effect and the postoperative analgesia effect. The results showed that compared with other algorithms, the evaluation index of ultrasound images processed by the 3D reconstruction algorithm was better. In terms of anesthesia effect, there was no significant difference in systolic blood pressure, diastolic blood pressure, and heart rate between the two groups before surgery (*P* > 0.05). Intraoperative and postoperative indicators of the experimental group were significantly better than those of the control group; the drug dosage (61 mg) was less than that of the control group (78 mg). In addition, the onset time of anesthesia, the time of pain blockade, and the postoperative awake time (5 minutes, 8 minutes, and 8 minutes, respectively) were shorter than those in the control group (13 minutes, 15 minutes, and 15 minutes, respectively). The visual analogue scale (VAS) scores of the experimental group were better than those of the control group on the day after surgery, one day after surgery, two days after surgery, and three days after surgery, with significant differences (*P* < 0.05). In summary, 3D reconstruction algorithm-based ultrasound image effect was clearer, the effect of UG-SNBA was more stable, and the postoperative analgesic effect was better. This work provided a higher reference for the selection of safe and effective anesthesia options in orthopedic surgery.

## 1. Introduction

Orthopedic surgery is clinically divided into four levels, ranging from simple to complex. The first-level surgery mainly refers to debridement, and the second-level surgery mainly refers to traumatic tendon repair. The third-level surgery mainly refers to complicated internal fixation of limbs, bone shaft fractures, and intra-articular fractures, and the fourth-level surgery mainly refers to the surgery of the cervical spine [1, 2]. The elderly are the main patients suffering from orthopedic diseases, especially the lower limb bones. The main reason is that with age, the loss of calcium in the body leads to osteoporosis, which makes the incidence of orthopedic diseases in the elderly dramatically higher than patients of other ages. For the elderly patients during orthopedic surgery, more requirements are required during the surgery due to their weaker functions in all aspects of the body, so that the anesthesia effect of the elderly patients can be more secure in surgery [3, 4].

When elderly patients undergo anesthesia surgery on the lower extremities, sciatic nerve block anesthesia (SNBA) is generally performed, which is one of the local anesthesia. The principle of nerve block anesthesia is described as follows. The local anesthesia drug was injected near the peripheral nerve trunk to block the conduction of nerve impulses, thereby making this part of the nerve controlled area anesthesia [5]. The sciatic nerve is composed of the fourth lumbar to the three anterior branches of the sacrum and is the largest body nerve. It ranges from the foramen of the piriformis muscle out of the pelvis, goes to the deep surface of the gluteus maximus, then passes through the greater trochanter and ischial tuberosity, and then, descends to the back of the thigh, which mainly affects the calf and foot. When the SNBA is adopted, the puncture point is often used between the piriformis muscle and the superior muscle. There are two methods of anesthesia, namely, the lateral position sciatic nerve block method and the supine position sciatic nerve block method [6, 7]. In anesthesia, the anesthesia teacher usually finds a suitable puncture location based on his own past experience. However, due to the large differences in the body of elderly patients, there are different signs on the body surface, which makes the difficulty of puncture success increase, decreasing the success rate of anesthesia. The introduction of ultrasound technology to assist anesthesia in orthopedic surgery can improve the success rate of puncture and make the anesthesia effect better [8].

Ultrasound technology to guide the nerve tissue is a new and innovative technology. Ultrasound interacts with human tissue to form information and then enlarges the information [9] to form an image, which is used to determine the specific location of human tissue, so as to assist doctors in better treatment of patients [10]. Due to the low time efficiency of traditional ultrasound technology, the image quality is relatively unclear. With the development of information technology, modern medical imaging technologies such as computed tomography and ultrasound have also developed. Compared with other imaging technologies, ultrasound is less harmful to the human body, and the speed of ultrasound imaging is faster. In addition, it shows the characteristics of real-time, which can give the doctor a timely response to the patient's tissue location and pathology [11, 12]. On this basis, great progress has been made in medical diagnosis and treatment technology. However, two-dimensional (2D) images can only express the anatomical information of a certain section and cannot determine the three-dimensional (3D) structure of the tissue and the relationship between them. Therefore, it is necessary to display the 3D structure and shape of human organs and obtain structural information that cannot be provided by traditional methods [13]. The 3D reconstruction algorithm of medical images can convert 2D images into 3D images with intuitive 3D effects, showing the 3D shape of human tissue. The region of interest can be observed from multiple directions and angles to obtain more information, which is of great significance for clinicians to formulate more scientific surgical plans [14, 15]. The introduction of the ultrasound-guided nerve block of the intelligent 3D reconstruction algorithm in the anesthesia during orthopedic surgery can better assist in the orthopedic surgery. There have been many reports on the ultrasound image of 3D reconstruction algorithm, but there are few studies on its application to guided nerve block in orthopedic surgery anesthesia and postoperative analgesia effect. In this study, the role of ultrasound-guided SNBA (US-SNBA) based on the intelligent 3D reconstruction algorithm in orthopedic surgery anesthesia and postoperative analgesia effect was explored, aiming to provide a theoretical guidance for clinical orthopedic surgery.

## 2. Materials and Methods

### 2.1. Objects and Grouping

In this study, 68 elderly patients who underwent orthopedic surgery on the lower extremities in hospital from January 2019 to January 2020 were selected as subjects, including 36 males and 32 females. The patients who did not cooperate in the whole process in the later period were excluded. They were randomly divided into two groups, with 34 people in each group. Subjects in the experimental group were 20 males and 14 females, and there were 16 males and 18 females in the control group. The patients in control group received sciatic nerve block anesthesia (SNBA), and those in the experimental group received ultrasound-guided SNBA (UG-SNBA) under 3D reconstruction algorithm to analyze and compare the anesthesia effect and the postoperative analgesia effect. This study had been approved by ethics committee of the hospital. The patients and their families had signed the relevant informed consents.

Inclusion criteria are as follows: the age range was between 60 and 80 years old; the patients were clinically diagnosed to be able to undergo orthopaedic surgery; and the patients had not undergone other surgical treatment recently.

Exclusion criteria are as follows: patients with other organic diseases, patients with incomplete clinical data acquisition, and patients who did not cooperate with the whole treatment.

### 2.2. Principles of 3D Reconstruction Algorithm

3D reconstruction is the main purpose of human vision and the main research direction of computer vision. It represents the process of recovering the 3D coordinates of spatial points from a single image plus scene constraints and two or more images (Figure 1).

3D reconstruction requires depth measurement. Firstly, the depth information of the object or scene was obtained, and then, the 3D modeling was performed to form a 3D representation of the object or scene. The flowchart was shown in Figure 2 below.

3D scene reconstruction includes surface reconstruction and weight reconstruction. Surface reconstruction describes the 3D structure of the object through the splicing of geometric units to fit the surface of the object. There are polygonal mesh surfaces, curved surfaces, tensor product surfaces, and superquadric. The surface patch was expressed by a polynomial, and the plane was shown in Equation (1); the bilinear surface, hyperboloid patch, bicubic surface, and subsurface patch were shown in Equations (2)–(5), respectively. In the below equations, *Z* was the surface patch, *a* referred to the coefficient, and *x* and *y* represented the coordinate axes.

(1) $$\begin{array}{c} Z_{1}=a_{0}+a_{1}x+a_{2}y, \end{array}$$

(2) $$\begin{array}{c} z_{3}=z_{2}+a_{4}x^{2}+a_{5}y^{2}, \end{array}$$

(3) $$\begin{array}{c} z_{2}=z_{1}+a_{3}xy, \end{array}$$

(4) $$\begin{array}{c} z_{4}=z_{3}+a_{6}x^{3}+a_{7}x^{2}y+a_{8}xy^{2}+a_{9}y^{3}, \end{array}$$

(5) $$\begin{array}{c} z_{5}=z_{4}+a_{10}x^{4}+a_{11}x^{3}y+a_{12}x^{2}y^{2}+a_{13}xy^{3}+a_{14}y^{4}. \end{array}$$

For triangular surface interpolation, the image plane coordinates were calculated for a point (*a*, *b*) in the image, and the *x* coordinate and *y* coordinate were expressed in Equation (6) and Equation (7), respectively.

(6) $$\begin{array}{c} x_{b}=b-\frac{m-1}{2}, \end{array}$$

(7) $$\begin{array}{c} y_{a}=-a+\frac{n-1}{2}. \end{array}$$

The three noncollinear points of the store in the depth image were obtained, and the plane corresponding to the three points were calculated. The depth value of (*a*, *b*) on the plane was calculated with

(8) $$\begin{array}{c} z_{ab}=a_{0}+a_{1}x_{b}+a_{2}y_{a}. \end{array}$$

When a 3D image was constructed, its linear interpolation can be used to model the surface patch through a binary linear function, as shown in

(9) $$\begin{array}{c} f\left(x,y,z\right)=a_{0}+a_{1}x+a_{2}y+a_{3}z+a_{4}xy+a_{5}yz. \end{array}$$

The minimum median square rule and the resampling strategy were adopted to achieve robust regression, as shown in Equation (10), in which *c* and *a* in the above equation both represented coefficients.

(10) $$\begin{array}{c} \text{argmin}\left|\text{med}\left[z_{a}-f\left(x_{a},y_{b}\right);c\right]\right|. \end{array}$$

When the surface was approximated, the model of the reconstructed surface was set as

(11) $$\begin{array}{c} z=f\left(x,y;a_{0},a_{1},\cdots a_{m-1}\right). \end{array}$$

The surface reconstruction is actually a regression of determining the parameters of the surface model for the most suitable data. The regression function was shown in

(12) $$\begin{array}{c} \chi^{2}=\overset{n-1}{\underset{a=0}{\sum }}\left(z-f{\left(x,y;a_{0},a_{1},\cdots a_{m-1}\right)}^{2}\right). \end{array}$$

When the function was regularized, an approximation constraint function can be added to make the surface you selected, and there was a unique solution for the function, as shown in

(13) $$\begin{array}{c} \chi^{2}=\overset{n-1}{\underset{a=0}{\sum }}\left(z_{a}-f{\left(x_{a},y_{b}\right)}^{2}+\alpha^{2}\iint \left(\frac{\partial^{2}f}{\partial x^{2}}+2\frac{\partial f}{ax}\frac{\partial f}{ay}+\frac{\partial^{2}f}{\partial y^{2}}\right)dxdy\right). \end{array}$$

The result of the trilinear interpolation was shown in Equation (14), and the isosurface was defined as Equation (15), in which *c* was a constant.

(14) $$\begin{array}{c} f\left(x,y,z\right)=a_{0}+a_{1}x+a_{2}y+a_{3}z+a_{4}xy+a_{5}yz+a_{6}zx+a_{7}xyz, \end{array}$$

(15) $$\begin{array}{c} \left(x,y,z\right)\left|f\left(x,y,z\right)=c\right.. \end{array}$$

### 2.3. Surgical Procedure

For all patients, it should establish intravenous access, closely monitor the vital signs, intravenously inject 0.5 mg penehyclidine hydrochloride injection, and take nerve block anesthesia after anesthesia induction took effect. The control group was anesthetized by sciatic nerve block under the guidance of nerve stimulator. Using the midpoint of the line connecting the most prominent part of the ischial tubercle and the greater trochanter of the femur as the puncture point, the 21 G puncture needle was vertically pierced into the skin. The current of the nerve stimulator was adjusted to 1.0 mA, and the current was adjusted to 0.4 mA after the motor response of the peroneal or tibial nerve was generated. In addition, it should inject 20 mL of 0.4% acid ropivacaine injection.

The research group performed ultrasound-guided sciatic nerve block anesthesia. The patient was placed in the lateral decubitus position, and ultrasound probe was placed between the femoral tubercle and the greater trochanter in the subgluteal region and was closely attached to the lower part of the gluteal groove and perpendicular to the long axis of the thigh. The direction of the probe was adjusted, and the sciatic nerve was identified in the hyperechoic greater trochanter, between the ischial tuberosity, deep gluteus maximus, and between the quadratus femoris, and showed a hyperechoic honeycomb image. A 21 G puncture needle was used to insert the needle in the plane to the side of the sciatic nerve, and then 20 mL of 0.4% ropivacaine was injected to complete the block anesthesia.

### 2.4. Image Evaluation Indicators

For the effect evaluation of ultrasound images, peak signal-to-noise ratio (PSNR) and structural similarity (SSIM) were used. PSNR was a measure of image quality and was often expressed in logarithmic decibel (dB) units. The calculation of PSNR first needed to know the calculation of mean square error (MSE). It was assumed that two *m* × *n* monochrome images were *I* and *K*, if one was similar to the noise of the other, then its MSE was defined as follows:

(16) $$\begin{array}{c} \text{MSE}=\frac{1}{mn}\overset{m-1}{\underset{i=0}{\sum }}\overset{n-1}{\underset{j=0}{\sum }}{\left[I\left(i,j\right)-K\left(i,j\right)\right]}^{2}. \end{array}$$

MSE was a common loss function, and PSNR was obtained through MSE. The equation was as follows:

(17) $$\begin{array}{c} \text{PSNR}=10∙\log_{10}\left(\frac{{\text{MAX}}_{I}^{2}}{\text{MSE}}\right)=20∙\log_{10}\left(\frac{{\text{MAX}}_{I}}{\sqrt{\text{MSE}}}\right). \end{array}$$

PSNR higher than 40 dB indicated that the image quality was excellent, that is, very close to the original image. 30-40 dB usually indicated good image quality (i.e., distortion is perceptible but acceptable), 20-30 dB indicated poor image quality; and PSNR below 20 dB indicated unacceptable image quality.

SSIM was an indicator that measures the similarity of two pictures and was often used for the evaluation of image quality. The input of SSIM was two images. It was assumed that the two input images were *x* and *y*, respectively, and the equation was as follows:

(18) $$\begin{array}{c} \text{SSIM}\left(x,y\right)={\left[l\left(x,y\right)\right]}^{\alpha }{\left[c\left(x,y\right)\right]}^{\beta }{\left[s\left(x,y\right)\right]}^{\gamma }. \end{array}$$

In the above equation, *l*(*x*, *y*) referred to the brightness comparison, *c*(*x*, *y*) was the contrast comparison, and *s*(*x*, *y*) was the structural comparison. SSIM was a number between 0 and 1. The larger the value, the smaller the gap between the output image and the undistorted image, that is, the better the image quality.

### 2.5. Observation Indicators

The difference between the ultrasound image under the 3D reconstruction algorithm and the traditional image was compared and analyzed, and then, the systolic blood pressure (SBP), diastolic blood pressure (DBP), and heart rate of the experimental group and the control group were compared before, during, and after the surgery. When the anesthesia effect was analyzed, the drug dosage, anesthesia onset time, pain block time (PBT), and postoperative wakefulness time (PWT) were compared between the two groups. After the surgery, the effect of postoperative analgesia effect was analyzed using the visual analogue scale (VAS). The VAS scoring criteria were shown in Figure 3. 0-2 means “comfortable,” 3-4 means “mild discomfort,” 5-6 means “moderate discomfort,” 7-8 means “severe discomfort,” and 9-10 means “extremely discomfort.”

### 2.6. Statistical Methods

The data of this experimental study was analyzed and processed using SPSS 19.0 version statistical software. The measurement of the data was expressed in the form of the mean ± standard deviation ($\bar{x}\pm s$), and the analysis of the count data was expressed by the percentage (%). The pairwise comparison between the data was realized using analysis of variance. *P* < 0.05 indicated that the difference was statistically significant.

## 3. Results

### 3.1. Ultrasound Images under 3D Reconstruction Algorithm

The following were two typical cases. Patient A, male, 60 years old, underwent internal fixation of a tibial fracture and underwent ultrasound-guided sciatic nerve + common peroneal nerve block. Patient B, male, 54 years old, underwent unilateral below-knee surgery with ultrasound-guided sciatic nerve + femoral nerve block.  Figure 4 showed ultrasound images of two patients.

Because it was necessary to determine the position of the surrounding blood vessels during the lower limb bone surgery, Figure 5 showed the blood vessel ultrasound image of three random patients. The blood vessel image near the lower limb bone under the ultrasound guidance of the intelligent 3D reconstruction algorithm showed clearer image.

### 3.2. Comparison of Processing Effects of Different Algorithms

The effect of the algorithm applied in this work was compared with that of BM3D, DnCNN, and Red-Net algorithms. As shown in Table 1, the PSNR and SSIM of the 3D reconstruction algorithm were better than other algorithms, and the difference was significant (*P* < 0.05).

### 3.3. Comparison on SBP, DBP, and Heart Rate

As shown in Figure 6, the SBPs were 135 ± 5.67 mmHg, 138 ± 5.27 mmHg, and 141 ± 5.87 mmHg for three preoperative measurements, 120 ± 4.89 mmHg, 124 ± 4.86 mmHg, and 119 ± 4.37 mmHg for three intraoperative measurements, and 129 ± 6.35 mmHg, 131 ± 6.64 mmHg, and 133 ± 6.26 mmHg for three postoperative measurements in the experimental group. The SBPs were 137 ± 6.38 mmHg, 139 ± 6.45 mmHg, and 136 ± 6.32 mmHg for three preoperative measurements; 130 ± 5.03 mmHg, 129 ± 5.25 mmHg, and 128 ± 5.28 mmHg for three intraoperative measurements; and 149 ± 5.98 mmHg, 151 ± 5.86 mmHg, and 143 ± 5.15 mmHg for three postoperative measurements.

As shown in Figure 7, the DBPs were 89 ± 2.37 mmHg, 87 ± 2.48 mmHg, and 91 ± 2.74 mmHg for three preoperative measurements; 80 ± 2.74 mmHg, 84 ± 2.69 mmHg, and 81 ± 2.85 mmHg for three intraoperative measurements; and 87 ± 3.06 mmHg, 88 ± 3.05 mmHg, and 86 ± 3.14 mmHg for three postoperative measurements in the experimental group. The DBPs were 93 ± 2.48 mmHg, 87 ± 2.86 mmHg, and 89 ± 2.57 mmHg for three preoperative measurements; 68 ± 2.46 mmHg, 71 ± 2.63 mmHg, and 73 ± 2.74 mmHg for three intraoperative measurements; and 96 ± 3.33 mmHg, 92 ± 3.26 mmHg, and 95 ± 3.37 mmHg for three postoperative measurements.

As shown in Figure 8, the three preoperative heart rate measurements were 81 ± 3.36 beats/sec, 80 ± 3.67 beats/sec, and 77 ± 3.84 beats/sec; the intraoperative measurements were 75 ± 4.02 beats/sec, 73 ± 4.04 beats/sec, and 76 ± 4.24 beats/sec; and the postoperative measurements were 77 ± 4.68 times/second, 79 ± 4.74 times/second, 78 ± 4.23 times/second, respectively. The heart rate of the patients in the control group was measured three times, and the values were 80 ± 3.47 beats/sec, 79 ± 3.75 beats/sec, and 76 ± 3.55 beats/sec before the surgery; 69 ± 3.97 beats/sec, 71 ± 3.79 beats/sec, and 68 ± 3.85 beats/sec during the surgery; and 87 ± 3.98 times/sec, 88 ± 3.74 times/sec, and 85 ± 3.64 times/sec after the surgery.

In Figure 9, P1, P2, and P3 referred to preoperative, intraoperative, and postoperative, respectively; (a–c) patient's SBP, DBP, and heart rate, respectively. The average values of SBP measured before, during, and after the surgery of the experimental group were 138 ± 6.46 mmHg, 121 ± 6.36 mmHg, and 131 ± 6.63 mmHg, respectively, while those in the control group were 137 ± 6.24 mmHg, 129 ± 6.85 mmHg, and 148 ± 6.47 mmHg, respectively. The average values of DBP measured before, during, and after the surgery were 89 ± 5.47 mmHg, 81 ± 5.94 mmHg, and 87 ± 5.25 mmHg of the experimental group, respectively, while those were 90 ± 5.24 mmHg, 71 ± 5.83 mmHg, and 94 ± 5.27 mmHg in the control group. The average heart rate values measured before, during, and after the operation were 79 ± 4.36 beats/sec, 75 ± 4.86 beats/sec, and 78 ± 4.95 beats/sec in the experimental group and 78 ± 4.45 beats/sec, 69 ± 4.58 beats/sec, and 87 ± 4.69 beats/sec in the control group, respectively. The differences between the two groups before surgery were not remarkable (*P* > 0.05), but they were statistically obvious during and after the surgery (*P* < 0.05).

### 3.4. Intraoperative Anesthesia Effect

When the anesthesia effect was analyzed, the average drug dosage of the experimental group was 61 ± 2.78 mg, and that in the control group was 78 ± 2.65 mg (as shown in Figure 10(a)). As illustrated in Figure 10(b) below, the average anesthesia onset time, the average PBT, and the average PWT of patients in the experimental and control groups were 5 ± 1.35 minutes vs. 13 ± 1.65 minutes, 8 ± 1.64 minutes vs. 15 ± 1.47 minutes, and 8 ± 1.68 minutes vs. 15 ± 1.64 minutes, respectively. Therefore, the differences between two groups were obvious statistically (*P* < 0.05).

### 3.5. Postoperative Analgesia Effect

The average VAS scores of the two groups were compared within three days after operation, and the results were given in Figure 11. The VAS scores in experimental group and the control group were 0.8 ± 0.45 and 3.3 ± 0.68 on the day of surgery, 2.5 ± 0.32 and 4.9 ± 0.85 on the day after surgery, 1.5 ± 0.24 and 3 ± 0.47 on the two days after surgery, and 1.3 ± 0.53 and 2.3 ± 0.74 on the three days after surgery, showing statistically notable differences (*P* < 0.05).

## 4. Discussion

Elderly patients have poor body tolerance; the function of various organs declines and often accompanied by a variety of underlying diseases. In this case, clinical lower extremity fracture surgery is performed, so there is a higher requirement for intraoperative anesthesia [16]. Traditional orthopedic surgery anesthesia mostly uses general anesthesia, which is convenient for ventilation and management, so it is widely used in clinical practice. However, intubation and extubation may increase myocardial oxygen consumption, increase heart rate and blood pressure, and increase the cardiovascular burden of patients [17]. The key to nerve block anesthesia is nerve positioning. The nerve stimulation needle is accurately placed near the target nerve, which can reduce the damage to nerves and blood vessels, and the anesthesia effect can be fully exerted. Nerve stimulator belongs to the traditional anatomical positioning method of nerve block anesthesia. Although the positioning is accurate, it requires high operator skills and experience. Otherwise, it is difficult to identify the diffusion of anesthetics and affect the blocking effect [18]. In recent years, with the development of ultrasound technology, its application in internal medicine has become more and more extensive, which also provides support for the application in the anatomical positioning of nerve block anesthesia. Using ultrasound guidance, not only can accurately locate but also facilitate the observation of drug diffusion [19].

In this work, the intelligent 3D reconstruction algorithm was used to optimize the ultrasound, and at the same time, it was used as a guide for nerve block in the orthopedic surgery of elderly patients in the control group and the experimental group. In addition, the effect of anesthesia and postoperative analgesia was analyzed. The results showed that the ultrasonic image evaluation index (PSNR: 35.216 and SSIM: 0.853) of the intelligent 3D reconstruction algorithm was better than other algorithms. After ultrasound guidance, according to the observation records, there was no significant difference in the systolic blood pressure, diastolic blood pressure, and heart rate between the two groups before operation. The indexes of the experimental group during operation and after operation were better than those of the control group (*P* < 0.05), and the anesthesia effect was more stable. This is consistent with the results of Li et al. [20]. The position of the sciatic nerve is shallow, and the algorithm-optimized ultrasound guidance can clearly display the target nerve structure, as well as the local drug diffusion, observe the path of the nerve stimulation needle, avoid nerve damage, and improve the effect of nerve block anesthesia. The drug dosage of the experimental group (61 mg) was also less than that of the control group (78 mg). The onset time of anesthesia, pain block time, and postoperative awakening time (5 minutes, 8 minutes, and 8 minutes) were all shorter than those of the control group (13 minutes, 15 minutes, and 15 minutes). The VAS scores of the experimental group were better than those of the control group on the day after surgery, one day after surgery, two days after surgery, and three days after surgery, with significant differences (*P* < 0.05). This point was also mentioned in the article of Selame et al. [21]. The application of ultrasound guidance in sciatic nerve block anesthesia can improve the safety of the block and the success rate of the block. Because the application of the nerve stimulator has a certain blind spot, it is difficult to observe the target nerve and drug diffusion. Ultrasound-guided nerve block anesthesia can observe the scope of drug injection in real time and make timely adjustments to ensure the effect of anesthesia. This anesthesia method can also effectively avoid nerve and blood vessel damage. Therefore, it is necessary to pay attention to the design of anesthesia plan in the process of lower extremity fracture surgery, so as to reduce the impact on the patient's breathing and blood circulation and improve the success rate and safety of anesthesia.

## 5. Conclusion

In this study, ultrasound-guided nerve block anesthesia based on three-dimensional reconstruction algorithm was used to analyze the effect of anesthesia and postoperative analgesia. The results showed that the ultrasonic images processed by the algorithm were clearer, and the anesthesia effect of orthopedic surgery under the guidance of the algorithm was more stable and obvious, and the analgesic effect was stronger. The disadvantage was that the patient sample in this work was small, and the experimental results would be biased in this case. Therefore, the selection of sample size should be increased in future experimental research, and the anesthesia and postoperative analgesia effects of ultrasound-guided nerve block based on 3D reconstruction algorithm in orthopedic surgery should be further analyzed and compared. In conclusion, this study provides data support and theoretical basis for the anesthesia scheme of clinical orthopedic surgery.

## Figures and Tables

**Figure 1:** Schematic diagram of image reconstruction.

**Figure 2:** Flow chart of 3D reconstruction.

**Figure 3:** The VAS scoring criteria.

**Figure 4:** The traditional ultrasound images. (a) Fibula is marked in orange and tibia in green; (b) Femur is shown in blue.

**Figure 5:** The blood vessel ultrasound images under intelligent 3D reconstruction. (a–c) The blood vessel images of three random patients, respectively.

**Figure 6:** Comparison on SBP of patients in two groups. (a–c) The SBP values before, during, and after the surgery, respectively.

**Figure 7:** Comparison on DBP of patients in two groups. (a–c) The DBP values before, during, and after the surgery, respectively.

**Figure 8:** Comparison on heart rate of patients in two groups. (a–c) The heart rates before, during, and after the surgery, respectively.

**Figure 9:** Comparison on different parameters of patients in different groups. (a–c) The comparisons of SBP, DBP, and heart rate, respectively. ^∗^Compared with control group, *P* < 0.05.

**Figure 10:** Comparison on intraoperative anesthesia effect. (a) The comparison on average drug dosage; (b) the comparisons on anesthesia onset time, PBT, and PWT, respectively. ^∗^Compared with control group, *P* < 0.05.

**Figure 11:** Comparison on VAS scores of patients in different groups. ^∗^Compared with control group, *P* < 0.05.

**Table 1:** Comparison of the effects of different algorithms.

Algorithm	PSNR (dB)	SSIM (dB)
BM3D algorithm	24.374	0.587
DnCNN algorithm	30.287	0.638
Red-Net algorithm	29.498	0.737
3D reconstruction algorithm	35.216^∗^	0.853^∗^

^∗^Compared with other algorithms, *P* < 0.05.

## Data Availability

The data used to support the findings of this study are available from the corresponding author upon request.
